# Identifying Animals in Camera Trap Images via Neural Architecture Search

This article has been retracted.

**DOI:** 10.1155/2022/8615374

**Published:** 2022-02-07

**Authors:** Liang Jia, Ye Tian, Junguo Zhang

**Affiliations:** ^1^School of Technology, Beijing Forestry University, Beijing 100083, China; ^2^School of Microelectronics and Control Engineering, Changzhou University, Changzhou 213164, China

## Abstract

Wild animals are essential for ecosystem structuring and stability, and thus they are important for ecological research. Since most wild animals have high athletic or concealable abilities or both, it is used to be relatively difficult to acquire evidence of animal appearances before applications of camera traps in ecological researches. However, a single camera trap may produce thousands of animal images in a short period of time and inevitably ends up with millions of images requiring classification. Although there have been many methods developed for classifying camera trap images, almost all of them follow the pattern of a very deep convolutional neural network processing all camera trap images. Consequently, the corresponding surveillance area may need to be delicately controlled to match the network capability, and it may be difficult to expand the area in the future. In this study, we consider a scenario in which camera traps are grouped into independent clusters, and images produced by a cluster are processed by an edge device installed with a customized network. Accordingly, edge devices in this scenario may be highly heterogeneous due to cluster scales. Resultantly, networks popular in the classification of camera trap images may not be deployable for edge devices without modifications requiring the expertise which may be hard to obtain. This motivates us to automatize network design via neural architecture search for edge devices. However, the search may be costly due to the evaluations of candidate networks, and its results may be infeasible without considering the resource limits of edge devices. Accordingly, we propose a search method using regression trees to evaluate candidate networks to lower search costs, and candidate networks are built based on a meta-architecture automatically adjusted regarding to the resource limits. In experiments, the search consumes 6.5 hours to find a network applicable to the edge device Jetson X2. The found network is then trained on camera trap images through a workstation and tested on Jetson X2. The network achieves competitive accuracies compared with the automatically and the manually designed networks.

## 1. Introduction

Ecosystems in earth have irreplaceable ecological, societal, and economic value for human beings [1], but ecosystems can be compositionally and functionally changed by species extinctions [2], e.g., massive declines in large carnivore populations are likely to result in ecosystem instability [3], loss of large herbivores can alter ecosystems through the loss of ecological interactions [4], and digging mammals are vital for maintaining the ecosystem in Australia [5]. In ecosystems, some wild animals like vertebrates high up the food chain may affect many other plants and animal species low down the chain [3, 4]. To prevent their extinctions, wildlife research, protection, and management require reliable animal data, such as population distributions, trying not to disturb animals and their habitats. Traditional data acquisition means may not fully meet this requirement, e.g., radio collars, satellite-based devices, and airplane surveillance. With the development of automatic and information technologies, camera traps not only provide an effective solution to acquire animal data in a nonintrusive and remote manner [6] but also are suitable for detecting rare or secretive species [7]. Camera traps may produce millions of animal images requiring classification [8] which is commonly automated via machine learning or deep learning methods, especially through convolutional neural networks (CNNs) [9–16]. Although CNN-based methods are widely adopted in classifications, almost all methods are developed under the condition that all camera trap images are processed by a single network requiring intensive or even formidable computational resources, e.g., a high-performance computing cluster is employed to classify 3.3 M (million) camera trap images [15]. Consequently, the corresponding surveillance areas may need to be deliberately controlled to match the network capability, and it may be difficult to expand the area in the future.

One promising solution of establishing or expanding surveillance areas without limitations of CNN capabilities is grouping camera traps as clusters accompanied by edge devices installed with customized CNNs [16, 17]. Thus, the computationally intensive classification of all images could be divided into subclassifications and offloaded to edge devices. Accordingly, edge devices may be highly heterogeneous [18] due to the cluster scales. Consequently, CNNs popular in classifications of camera trap images might not be deployable for edge devices without modifications such as quantization, pruning, and neural network design [19]. Among these modifications, neural network design significantly improves the computation and storage efficiency of CNN [19], but “designing neural networks is very difficult, and it requires the experience and knowledge of experts, a lot of trial and error, and even inspiration” [20]. Fortunately, the design can be automated by neural architecture search (NAS) [21–28].

With advancements in NAS, it is practical and automatic to design CNNs with performances competitive with ones designed by human experts [21–28]. However, the automatic design via NAS may be tough due to the dimension explosion of search space and the expensive evaluations of candidate networks. Since the search space is defined with respect to (w. r. t.) the meta-architecture, i.e., the prototype from which the candidate networks are developed, a lot of effort has gone into reducing the structure complexity [28] of meta-architectures [21–27], e.g., high-dimensional chain architectures and low-dimensional cell architectures. The low dimensionality of the cell architecture arises from its repeatable local structures called cells [21–27]. The cell architecture is thus built by assembling cells sharing the same structure except weights. The network built on the chain architecture is equivalent to a single-cell network in view of the cell architecture. Therefore, the dimensionality of search space based on the cell architecture is much lower than the chain architecture. The dimensionality may further be reduced by simplifying cells.

There are two common types of cells, i.e., normal and reduction cells. Since the reduction cell mainly reduces data dimensions, the cell may be simplified to decrease the dimensionality of search space [24–27]. For instance, PNASNet [24] focuses on optimizing the normal cell only and implements the reduction cell by copying the normal cell and adjusting the convolution strides. Path-level network transformation [25] simplifies the reduction cell to a single pooling layer and models the normal cell as a tree. The search conducts a Net2DeeperNet operation to each node in the tree to change the cell topology. GDAS [27] optimizes normal cells only and adopts a manually defined reduction cell. However, meta-architectures are always fixed regardless of resources limited by edge devices [21–27].

These facts inspired us to develop a search method on the basis of an adaptive cell architecture that automatically changes w. r. t. resources restrained by devices [29]. The proposed method was designed within the framework of NAS based on reinforcement learning (RL) due to their good performances [22, 23, 30–32]. RL attempts to train an agent to perform actions to interact with the environment by receiving rewards based on the previous actions. Accordingly, the sampler (controller [22, 23]) learns from its sampled networks, especially the performances. However, the performance evaluation may be costly due to the expensive network training. The cost may be lowered by various means like minimizing training time [22] and sharing weights of trained networks during search [23]. After the search, the optimal network can either be selected from the search history [22, 30–32] or sampled by the trained sampler [23].

In this study, an RL-based search method is designed in consideration of resource-limited devices. Namely, the meta-architecture changes adaptively and automatically w. r. t. the resource limited by the device. Besides, the search is accelerated by predicting the test accuracy of the sampled networks through regression trees, i.e., the network structure is vectorized through conversion functions, and the resulting vectors are fed to regression trees to yield accuracy. On the basis of the search acceleration and the adaptive meta-architecture, a search method named neural architecture search based on regression tree (NASRT) is proposed in this study, and the main contributions are summarized as follows:

1. The proposed search method is designed in consideration of computational resources limited by edge devices for classifying camera trap images. This is achieved by using an adaptive meta-architecture that automatically changes w. r. t. the resource limit.
2. The proposed search method is accelerated by replacing the costly accuracy evaluation with economical prediction. This is achieved by vectorizing the sampled network and feeding the resulting vector to regression trees to estimate the accuracy.

The remainder of this study is organized as follows. In Section 2, NASRT is introduced. In Section 3, the test results of NASRT are shown and analysed. Finally, Section 4 gives the conclusion.

## 2. Methods

The flowchart of NASRT is shown in Figure 1 which highlights five steps of NASRT whose details are introduced sequentially in this section. As shown in the figure, long short-term memory (LSTM) [33] samples cell structures. The sampled cell is then assembled according to the adaptive meta-architecture w. r. t. resources limited by the edge device. The accuracy of the network is predicted by regression trees learned by XGBoost [34]. The predicted accuracy then serves as a component of reward which is employed to generate the loss to update the sampler LSTM.

The adaptive meta-architecture is depicted in Figure 2. The architecture consists of normal and reduction cells, i.e., tiny networks either preserving or halving data dimensions. In this study, every reduction cell is simplified to be a single pooling layer, and there are *R* reduction cells in total. For every two reduction cells, there are *N* normal cells. The cell pipeline terminates at the global average [35].

Obviously, adaptive meta-architecture can be built dynamically by changing values of *N* and *R* w.r.t. device-associated resources which are simplified as GPU memory ℳ in this study. Namely,

(1) $$\begin{array}{c} f=\begin{array}{cc} \underset{n=1\ldots N}{\max} & \left(\sum_{j=1}^{R}\left(\sum_{i=1}^{n}{\dot{C}}_{i}+{\ddot{C}}_{j}\right)+\sum_{i=1}^{n}{\dot{C}}_{i}\right),\\ \text{s.t}. & f<ℳ, \end{array} \end{array}$$

where *f* denotes the adaptive meta-architecture, *N* is the maximal number of normal cells between two consecutive reduction cells in *f*, *R* is a fixed constant referring to the total number of reduction cells in *f*, ${\dot{𝒞}}_{i}$ denotes the *i* th normal cell, ${\ddot{𝒞}}_{j}$ represents the *j* th reduction cell, “+” corresponds to the cell permutation in Figure 2, and “*f* < ℳ” denotes the resource constraint. Specifically, suppose the batch size (the number of images fed to the network at a time) and GPU memory for a specific application are known a priori, NASRT initializes the network based on formula (1) parameterized by *N* and attempts to load a single batch of data together with the network to GPU. If the loading fails because of insufficient GPU memory, the initialization and data loading will be repeated w. r. t. formula (1) parameterized by *N* − 1. This continues until the loading succeeds or *N* = 0 which will cause NASRT to abandon the current network.

As mentioned above, a normal cell is a tiny network, which means it has its own inner structure as shown in Figure 3. Even though normal cells share the inner structure in the same network, they differ in input sources and weights. The input sources are defined recursively. Namely, for the *i* th normal cell ${\dot{𝒞}}_{i}$ in Figure 3, input sources of a block are chosen from previous cells ${\dot{𝒞}}_{i-1}$, ${\dot{𝒞}}_{i-2}$ … ${\dot{𝒞}}_{i-B}$ (simplified to *𝒞*_−1_, *𝒞*_−2_ … in the followings). The choice is made by the sampler during the search. A block contains several operations, e.g., convolution and identity operations. The outputs of the operations within a block are collected and added to generate the block output, and the input of an operation can come from another block within the same cell or one of *B* previous cells.

There are five operations optional for a normal cell, i.e., *T*_3_^*c*^, *T*_5_^*c*^, *T*_3_^*d*^, *T*_5_^*d*^, and *T*^*I*^ where the first four operations denote stacks of convolution, batch normalization [36], and ReLU [37], and the last one denotes the identity operation. The convolution can be either depthwise separable [38] (*T*_3_^*d*^ and *T*_5_^*d*^) or not (*T*_3_^*c*^ and *T*_5_^*c*^), and its kernel size can be either 3-by-3 (*T*_3_^*d*^ and *T*_3_^*c*^) or 5-by-5 (*T*_5_^*d*^ and *T*_5_^*c*^). There are four pooling layers optional for a reduction cell, i.e., *T*_3_^*m*^, *T*_5_^*m*^, *T*_3_^*a*^, *T*_5_^*a*^. The pooling can be either max (*T*_3_^*m*^ and *T*_5_^*m*^) or average (*T*_3_^*a*^ and *T*_5_^*a*^), and its kernel size can be either 3-by-3 (*T*_3_^*m*^ and *T*_3_^*a*^) or 5-by-5 (*T*_5_^*m*^ and *T*_5_^*a*^).

The cells are sampled in step 1 of Figure 1. For each block in the normal cell, the number of its operations is selected from {2,  3 … *M*}. For each operation in a block, its type is chosen from {*T*_3_^*c*^, *T*_5_^*c*^, *T*_3_^*d*^, *T*_5_^*d*^, *T*^*I*^}, and its input is selected from {ℬ_−1_, ℬ_−2_…} or {*𝒞*_−1_,  *𝒞*_−2_…}, i.e., previous blocks or cells ({ℬ_−1_, ℬ_−2_…}=∅ for the first block). For the pooling layer in the reduction cell, the pooling is chosen from {*T*_3_^*m*^, *T*_5_^*m*^, *T*_3_^*a*^, *T*_5_^*a*^}, and its input is fixed to the previous cell. All the selections are made by the sampler LSTM based on its hidden states associated with the previous selections.

The network is built in step 2 of Figure 1 w. r. t. the adaptive meta-architecture defined by formula (1). During the building process, some steps require special attentions, e.g., for ${\dot{𝒞}}_{i}$ where 1 ≤ *i* < *B*, there are *i* previous cells instead of *B* cells. Especially for the first cell, only raw image data are available. In this case, the operation input is chosen from the available sources. When the inputs of operations in a block come from another block or cell, we call they are connected. Besides the input availability of an operation, its output is added with other operations within the same block, and this requires all the outputs to share the same dimension. Thus, downsampling is applied to outputs whose dimensions differ from the minimal one found within the block, and then, they are summed, i.e.,

(2) $$\begin{array}{c} {ℬ}_{j}=\sum_{k=1}^{m_{j}}T_{j,k}\left(I_{j,k}\right), \end{array}$$

where ℬ_*j*_ denotes the output of the *j*th block in a cell, *m*_*j*_ is the operation number, *I*_*j*,*k*_ represents the input of the *k*th operation *T*_*j*,*k*_. Among the blocks in a cell, there are ones not connected to any other blocks, and the outputs of these unconnected blocks are concatenated to yield the cell output ${\dot{𝒞}}_{i}$, i.e.,

(3) $$\begin{array}{c} {\dot{C}}_{i}=\underset{j^{*}}{⊕}{ℬ}_{j^{*}}\text{,}\\ \text{s.t}.\;{ℬ}_{j^{*}}\neq I_{j,k}\forall j,k, \end{array}$$

where the concatenation is denoted by ⊕. During concatenating the block outputs, upsampling is applied to the outputs whose dimension differs from the maximal one among the ones to concatenate.

The accuracy is predicted in step 3 of Figure 1 for a built network (all following steps will be skipped if the building fails at the GPU loading stage) through regression trees generated by XGBoost. Since the inputs of trees are vectors, the network needs to be vectorized. This requires selecting and scalarizing network components to generate a vector uniquely representing the network. In this study, normal cell structure, pooling layer type, the cell pipeline, and the channels of cell outputs are chosen as the components. For the pipeline, the expanded form of formula (1) is

(4) $$\begin{array}{c} f=\sum_{i=1}^{n}{\dot{C}}_{i}+{\ddot{C}}_{n+1}+\overset{2n+1}{\underset{i=n+2}{\sum }}{\dot{C}}_{i}+{\ddot{C}}_{2n+2}+\cdots +{\ddot{C}}_{Rn+R}+\sum_{i=R\left(n+1\right)+1}^{\left(R+1\right)n+R}{\dot{C}}_{i}.\; \end{array}$$

The pipeline is scalarized by

(5) $$\begin{array}{c} f_{s}=\sum_{C_{\ell }\in f}2^{\ell }\cdot \delta \left(C_{\ell }-\dot{C}\right), \end{array}$$

where *ℓ* corresponds to the cell index in formula (4) regardless of the cell type, the subtraction estimates whether the current cell is a normal cell $\dot{𝒞}$, and *δ*(*x*) is 1 if *x* is 0, and it is 0 otherwise. The output channels are scalarized by

(6) $$\begin{array}{c} Ch_{s}=\sum_{C_{\ell }\in f}\text{ch}\left(C_{\ell }\right), \end{array}$$

where the channel of the outputs yielded by *𝒞*_*ℓ*_ is denoted by ch(*𝒞*_*ℓ*_). The structure of the normal cell is scalarized w.r.t. each block, i.e.,

(7) $$\begin{array}{c} {\dot{B}}_{s,j}=\sum_{s\in S_{j}}{\text{idx}}_{S}\left(s\right)\cdot {\left|S\right|}^{{\text{idx}}_{S_{j}}\left(s\right)}, \end{array}$$

where *S*_*j*_={*I*_*j*,1_, *T*_*j*,1_ …  *I*_*j*,*m*_*j*__, *T*_*j*,*m*_*j*__} represents the structure of the *j* th block, i.e., the pairs of operation input and its type; *𝒮*={*T*_3_^*c*^, *T*_5_^*c*^, *T*_3_^*d*^, *T*_5_^*d*^, *T*^*I*^}+{*T*_3_^*m*^, *T*_5_^*m*^, *T*_3_^*a*^, *T*_5_^*a*^}+{ℬ_−1_, ℬ_−2_ … ℬ_−*B*+1_}+{*𝒞*_−1_,  *𝒞*_−2_ … *𝒞*_−*B*_} contains the inputs and types of operations available for sampling; idx_*S*_*j*__(*s*) finds the index of the member *s* from *𝒮*. Similarly, the pooling layer is scalarized as ${\ddot{B}}_{s}$. In short, the aforementioned formulae (5) to (7) are called conversion functions, and a given network *f* is vectorized by arranging the scalars yielded by the conversion functions, i.e.,

(8) $$\begin{array}{c} ℐ\left(f\right)=\left[\begin{array}{cc} \begin{array}{ccc} f_{s} & Ch_{s} & {\dot{B}}_{s,1} \end{array} & \begin{array}{ccc} \ldots & {\dot{B}}_{s,B} & {\ddot{B}}_{s} \end{array} \end{array}\right]. \end{array}$$

Since XGBoost is a supervised learning method, its training is based on datasets containing pairs of vectorized networks and their accuracies. The vector datasets are built by randomly sampling networks first and then training and validating sampled networks. The training and validation accuracies *A*_*T*_ and *A*_*V*_ together with the network result in two vector datasets: {vectors, *A*_*T*_ s} and {vectors, *A*_*V*_ s}. Two regression trees are built by XGBoost, respectively, based on the vector datasets. Thus, the training accuracy of a given network *f* is predicted by

(9) $$\begin{array}{c} A_{T}^{*}=T_{T}\left(ℐ\left(f\right)\right), \end{array}$$

and its validation accuracy is obtained similarly. The predicted accuracies are employed to generate a reward in step 4 of Figure 1, i.e.,

(10) $$\begin{array}{c} A=\max\left(0,\;\left(1-\alpha \right)A_{V}^{*}+\alpha \left(A_{V}^{*}-A_{T}^{*}\right)\right), \end{array}$$

where 0 < *α* < 1 is a hyperparameter. The definition of *A* differs from conventional rewards reported in NAS literatures [21–23]. This is because we noticed that the overfitting always occurs in the case that the validation accuracy does not improve while the training accuracy keeps high. Thus, to avoid networks easy to overfit, we introduced the difference between the training and the validation accuracies. Thus, if the validation accuracy is much smaller than the training accuracy, then the network may easily overfit, and the reward should be very low, which is reflected through *A* by a large negative value produced by the accuracy difference. However, we cannot have negative accuracies in practice; thus, we apply a ReLU function [37] to guarantee the resulting *A* is non-negative. The reward then serves to generate the loss *J*(*θ*) [39]:

(11) $$\begin{array}{c} J\left(\theta \right)=A\left(\sum_{j}^{B}\left(\log\left(P\left(n_{j}|\theta \right)\right)+\sum_{k}^{n_{j}}\log\left(P\left(a_{k}|a_{1\;:\;\left(k-1\right)},\theta \right)\right)\right)+\log\left(P\left(a|\theta \right)\right)\right), \end{array}$$

where *P*(*n*_*j*_*|θ*) denotes the probability of sampling the operation number *n*_*j*_ of the *j* th block in the normal cell, *P*(*a*_*k*_*|a*_1 : (*k* − 1)_, *θ*) is the probability of sampling the input and operation type for the *k* th block after the first (*k* − 1) operations have been sampled, and *P*(*a|θ*) represents the probability of sampling the operation for the reduction cell. The gradient ▽_*θ*_*J*(*θ*) is then employed for updating LSTM with weights *θ*.

In step 5 of Figure 1, the optimal network is selected from the search history w.r.t. specific requirements defined by the device. The networks filtrated by restrictions are decreasingly sorted by their rewards from search, and top 25% are retrained and tested w.r.t. a few epochs, e.g., 15 epochs. Then, the retrained networks are sorted according to their test accuracies, and top 25% are retrained and tested w.r.t. an increased epoch value. This repeats until one network is left, and this network serves as the output of the search.

## 3. Results and Discussion

The performances of NASRT are reflected by both the search efficiency and the performance of the resulting CNN. The search is based on CIFAR-10 [40]. The CNN performance is evaluated on wildlife datasets ENA24 [41] and MCTI [42]. The search efficiency of NASRT is compared with the classical and the state-of-art NAS methods, i.e., NASNet [22], PNASNet [24], PDARTS [43], SGAS [44], SETN [26], and MnasNet [45]. The CNN performance is compared with the manually derived networks Resnet-18 [46], DenseNet [47], and MobileNet-v2 [48] and the automatically designed networks PDARTS [24], SGAS [44], and SETN [26]. The hardware in experiments comprises Jetson X2 with NVIDIA Pascal GPU, a laptop with GeForce GTX 1060 GPU, and a server with four GPUs of NVIDIA TITAN Xp. The software of experiments involves CUDA 9.1, PyTorch 0.4.1, Python 3.6, and MySQL 8.

### 3.1. Datasets

There are three datasets employed in this study, i.e., CIFAR-10 [40], ENA24 [41], and MCTI [42]. These datasets serve for different purposes, i.e., CIFAR-10 serves for the search only, while datasets ENA24 and MCTI serve for classifying animal species. CIFAR-10 contains 60K 32-by-32 colour images categorized to ten classes in which six are animals, i.e., bird, cat, deer, dog, frog, and horse. ENA24 contains 8K 2048-by-1536 images categorized to 21 animal species including crow, cat, white-tailed deer, coyote to name a few. MCTI consists of 24K wildlife images whose resolutions range from 1920-by-1080 to 2048-by-1536, and the images are categorized into 20 wildlife species, e.g., bird, ocelot, roe deer, red fox. The and background habitats in camera trap images, the images of both ENA24 and MCTI are resized to 64-by-64. Obviously, some species from MCTI and ENA24 are closely related with some classes of CIFAR-10. The class relationship is graphically illustrated in Figure 4.

The testing images of either ENA24 or MCTI are randomly selected and account for 20% of all images of the corresponding datasets. For instance, there is a bear-shaped silhouette near the upper-left corner of the rectangle of ENA24 in Figure 4; at the foot of the silhouette, there is a label indicating the class name is black bear with 730 training and 163 testing images. The class relationship is visualized by rectangles expanded through datasets. Namely, if classes from different datasets are covered by the same rectangle, then either their shapes are similar or they are biologically related in taxonomy.

### 3.2. Search on CIFAR-10

Since over half classes of CIFAR-10 are animal species and most of the species are closely related to wildlife species shown in Figure 4, CIFAR-10 serves for finding CNN based on the adaptive meta-architecture as shown in Figure 2. The maximum values of normal cell number *N* and reduced cell number *R* are set to 5 and 3, respectively. The block number *B* and the operation number *M* are set to 5 and 4, respectively. For the combination of *R* = 3, *M* = 4, and *N* = *B* = 5, there are approximately 2.7 M candidate networks in the search space.

Regression trees are learned by XGBoost based on 0.02 M randomly sampled networks, and networks are selected so that their validation accuracies are evenly distributed. Specifically, the sampled networks are vectorized through conversion functions, trained on 40 K out of 50 K training images from CIFAR-10, and then validated on the left 10 K training images. Thus, the vectors and training accuracies, and the vectors and validation accuracies form two datasets to generate trees. Data augmentation of the training is the same as [23], and AMSGrad [49] serves as the optimizer whose learning rate is set to 0.005. The batch size is 128, and the epoch number is 1.

XGBoost involves twelve hyperparameters automatically determined by Bayesian optimization [50]. The details are introduced in Supplementary Materials (available here). Finally, 72 and 166 regression trees are generated by XGBoost, respectively, on training-accuracy-based and validation-accuracy-based vector datasets. The trees may be either shallow or deep as depicted in Figures 5 and 6, respectively.

For search, the hidden-unit number of LSTM is set to 300, and the dimension of word embedding is 512. The outputs of the softmax function serve as the probabilities of formula (11). AMSGrad serves as the optimizer of LSTM, and the learning rate is set to 10^−3^. The sampling times are 1.5 × 10^3^. The hyperparameter of formula (10) is set by *α*=0.4. Since randomness is inevitable in NAS, the searches are often repeated to obtain the optimal networks [21, 27]. Thanks to the proposed acceleration, the costs of repetitive searches are acceptable. Therefore, the search is repeated, until the result is considered satisfactory w.r.t. the resource limited by Jetson X2. Namely, the on-board memory of Jetson X2 is 8 GB which approximates 12 GB GPU memory of the workstation employed for search, but in Jetson X2, the memory is shared by both CPU and GPU. In experiments, we find that Jetson X2 memory available for GPU approximately corresponds to 5 GB of workstation, and then, this memory limit becomes the restriction to filtrate networks retrieved from the search history.

The normal cell of the optimal network found by NASRT is shown in Figure 7. In the figure, the operations are denoted by colour rectangles, the blocks are represented by dashed-line rectangles, and the cells are represented by rectangles with colourless faces and colour edges. The arrows indicate the connections among cells and blocks. There are *N*=3 normal cells in the pipeline of the resulting network, and 3-by-3 max pooling serves as the reduction cell. The channel number *d* throughout operations is set to 36, i.e., outputs of operations always have 36 channels. For operations altering channels, their hyperparameters are set to produce *d* output channels, e.g., the kernels of convolution, and for operations preserving channels, the channels of their inputs are mapped to *d* through a stack of the convolution with *d* kernels of size 1 × 1, batch normalization, and ReLU.

To evaluate the search efficiency, the search time of NASRT is compared with the classical and the state-of-art search methods, i.e., PDARTS, SGAS, SETN, PNASNet, MnasNet and NASNet-A, and the CNNs found by these methods are compared with the one of NASRT. The methods are compared w.r.t. the network parameter number in millions (“Para. (M)”), the inference time in seconds (“Test [sec.]”), GPU memory consumption in megabytes (“GPU (MB)”), and the search time in days when a single GPU is employed (“Time (GPU days)”) as shown in Table 1.

As shown in Table 1, the search time of NASRT, PDARTS, SGAS, and SETN is obtained by conducting the searches on our workstation with four Titan Xp GPUs. The search time of NASRT is the best throughout all methods, which validates its search efficiency. For the resulting network, its parameter number, inference time, and GPU memory consumption are obtained by feeding a 64-by-64 image to the network on the laptop of GTX 1060 GPU whose low computational capability specially serves the time estimation. In Table 1, NASRT consumes the second least GPU memory and the least search time.

### 3.3. Tests on ENA24

The CNN found by NASRT is tested on ENA24 to evaluate its performance in classifying animal species in camera trap images. The images in ENA24 are categorized to 21 species illustrated by the silhouettes in Figure 4 which also shows the number of the images serving for training and test. The CNN of NASRT is trained from scratch on training images. Before the training starts, the network parameters are initialized through Xavier uniform [51]. The data augmentation involves CutOut [52], horizontal image flip, image crop, and normalization. The CNN is optimized through stochastic gradient descent [53]. The learning rate is adjusted by a schedule of cosine [54] with hyperparameters *l*_max_=5 × 10^−3^ and *l*_min_=10^−1^. The batch size and epoch are set to 32 and 55, respectively.

Besides the proposed CNN, several manually derived and automatically derived CNNs are introduced in the experiments for comparison. The manually designed CNNs are Resnet-18, DenseNet, and MobileNet-v2. The automatically designed CNNs are SGAS, SETN, and PDARTS. These networks are trained based on the same configuration as NASRT with a smaller batch size due to their high consumptions of GPU memory as shown in Table 1. Accordingly, the batch sizes are set to 8 (SGAS, PDARTS) and 10 (SETN). However, the small batch requires more training time than the large batch, which means SGAS, SETN, and PDARTS will consume more computational resources than other methods if the epochs of all methods are the same. Hence, their epochs are halved to 25. The results are shown in Table 2 where the bold texts highlight the best accuracies for each row.

As shown in Table 2, the top three average accuracies are achieved by DenseNet (97.5%), NASRT (97.38%), and Resnet-18 (97.25%). The differences among the top three average accuracies are relatively small, while DenseNet and Resnet-18 are manually derived. Due to the decreased epoch numbers, SGAS (95.64%), SETN (94.15%), and PDARTS (95.94%) achieve the average accuracies lower than NASRT. For individual class accuracies, DenseNet achieves the best class accuracies for 14 classes, Resnet-18 for 12 classes, and NASRT for 10 classes. For NASRT, the bottom four class accuracies are associated with northern raccoon (94.12%), grey fox (94.67%), bobcat (95.16%), and cottontail (95.24%). To analyse the errors of NASRT, we start with the misclassifications of the general case as shown in Figure 8 and then continue with the bottom four accuracies as shown in Figures 9–12. In these figures, misclassified images and associated species predicted by NASRT with top five accuracies are illustrated, and the misclassified species and the correct species are, respectively, indicated with red and green colours.

As shown in Figure 8, the misclassification is made by NASRT when animals are blocked (left-most subfigure), of cryptic coloration (middle-left subfigure), blurred/night vision (middle-right subfigure), or partially visible in the images. The aforementioned cases may be overlapped as shown in Figures 9–12.

### 3.4. Tests on MCTI

The tests on ENA24 illustrate the performances of NASRT for limited data, i.e., there are totally 8K images for 21 species. It is curious to find out its performance under the contradictive condition, i.e., abundant data as in dataset MCTI (there are totally 24K images for 20 species). The training and testing on MCTI are the same as the case of ENA24, and the results are shown in Table 3.

As shown in Table 3, the top three average accuracies are achieved by NASRT (98.27%), SGAS (96.88%), and DenseNet (96.75%). The difference between the average accuracy of NASRT and any other network exceeds 1%. Among the manually derived networks, the average accuracy of Resnet-18 is very close to DenseNet, which may explain the popularity of Resnet-18 in wildlife identification [14, 15]. For individual class accuracies, NASRT outperforms all other networks throughout 16 species, even though there are still misclassifications made by NASRT. The typical misclassified images are shown in Figure 13, and the examples of three species with the lowest accuracies, i.e., ocelot (89.47%), red fox (95.6%), and red brocket deer (96.59%) are illustrated in Figure 14to 16. The fourth lowest accuracy is associated with a red squirrel (97.35%), and there are only two misclassified images, and one has been shown in Figure 13.

As shown in Figure 13, misclassification may occur when the animal is not side viewed (left-most subfigure), camouflaging (middle-left subfigure), blurred (middle-right subfigure), or partially visible (right-most subfigure). The aforementioned cases may overlap as shown in Figures 14–16.

### 3.5. Tests on Jetson X2

The previous sections illustrate the results of experiments conducted on the workstation with abundant computational resources. However, these experiments cannot illustrate the case of applying the proposed network to resource-constrained edge devices such as Jetson X2 as shown in Figure 17. Therefore, the network is retested on Jetson X2.

The software in experiments involves Ubuntu 18.06, Python 3.6.7, CUDA 10.0, Pytorch 1.1.0, and torchvision 0.2.0. Both the test images and the weights of the pretrained network are copied to Jetson X2 through secure copy protocol (SCP) in the local area network.  Table 4 shows the results from Jetson X2.

As shown in Table 4, the average accuracies of the proposed network are 97.03% and 98.23%, respectively, for datasets ENA24 and MCTI. The accuracies from Jetson X2 are slightly lower than the workstation (97.38% of ENA24 and 98.27% of MCTI).

## 4. Conclusions

In the present study, a neural architecture search method named NASRT is proposed for providing CNNs customized for diverse edge devices, and thus, edge devices can be incorporated with clusters of camera traps to set up or expand surveillance areas. There are mainly two challenges faced by NASRT, i.e., lowering search costs and searching networks feasible for edge devices. For the first challenge, the search costs are lowered by reducing the search space dimensionality and accelerating candidate network evaluations. The search space dimensionality is reduced by replacing the reduction cell with a single pooling layer, and the candidate network evaluation is accelerated via regression trees generated by XGBoost. Since regression trees can only process vectors, candidate networks are vectorized through conversion functions. For the second challenge, candidate networks are built w.r.t. an adaptive meta-architecture optimized according to computational resources defined by edge devices. On the basis of the simplified search space, the search acceleration, and the adaptive meta-architecture, NASRT successfully found a network applicable for the edge device Jetson X2, and its search time is the best in comparison. The performance of the network found by NASRT is evaluated on the data-limited dataset ENA24 and data-abundant dataset MCTI. The resulting average accuracies of identifying wildlife are, respectively, 97.38% and 98.27%, which are competitive compared with the classical and the state-of-art networks.

The limitations of the present study are mainly twofold, i.e., the benchmark dataset used in this study differs from the camera trap datasets in both the data distribution and the image aspectratio. For the first limitation, since surveillance areas of camera trap clusters may cover different habitats of wild animals, data distributions may differ from cluster to cluster. The present study employs a benchmark dataset named CIFAR-10 to search candidate networks, and thus, the architectures of the searched networks are optimized according to images from benchmark datasets instead of camera trap images. For the second limitation, the candidate networks in this study are assumed to process images with the aspect ratio 1 : 1, i.e.., images with the same widths and heights, as other CNNs popular in the classification of camera trap images. However, camera trap images are usually 4 : 3 as shown in the section of results. The assumption of aspect ratio 1 : 1 requires images to be resized, and there are mainly two means to resize an image, i.e., rescaling the image without maintaining its original aspect ratio or padding short edges of the image to maintain its original aspect ratio. The former results in deformed animals, and the latter introduces interpolated pixels. Neither misshaped animals nor interpolated pixels would be helpful for the classification.

Future work mainly concerns the application of camera trap images in the search, i.e., searches are conducted directly on camera trap images rather than images from benchmark datasets. Since camera trap images differ from benchmark dataset images in many aspects, especially the aspect ratios, a preprocessing step is expected to be developed to maintain the aspect ratios of camera trap images. Moreover, differences among images from different types of camera traps need to be considered in future studies.

## Figures and Tables

**Figure 1:** Flowchart of the proposed method named NASRT, This figure illustrates the main steps of NASRT where the first four steps represent the procedure of a single sampling during the search, and the search commonly repeats the sampling multiple times. Once the search ends, the optimal network is selected from the search history as indicated by step five in the figure.

**Figure 2:** Adaptive meta-architecture of NASRT. The meta-architecture determines how a candidate network is built during the search and how the data flow through the network. The data flow from the input to the output via multiple paths in a candidate network, and paths are dynamically determined by the sampler during the search. The dynamic paths are represented by both a cloud shape labelled “cell connection” and lines emitting from it. Candidate networks building is affected by several user-defined constants, e.g., normal cell number *N* and reduction cell number *R*, respectively, denoted by “*N*” and “…” in the figure.

**Figure 3:** Inner structure of a normal cell in a candidate network. This figure illustrates the inner structure of the *i* th normal cell denoted by a large rectangle with the upper-left corner labelled “cell *i*”. A normal cell consists of operations grouped as blocks, and there are *B* blocks represented by smaller rectangles with upper-left corners labelled “block 1” … “block *B*”. The number of operations in a block is dynamically determined by the sample during the search, and this dynamic number is represented by “…” between two operations in each block. The input of an operation is also dynamically determined by the sampler, and the input is usually sampled from previous cells or blocks, which means outputs of cells or blocks may serve as operation inputs. The cell output is denoted by an arrow emitting from the cell, and an operation output is represented by an arrow emitting from the operation. Outputs of operations not serving as inputs of any other operations are summed to yield the block output, the sum is represented by a rectangle labelled “add”, and the block output is denoted by an arrow emitting from the rectangle. The input and output relationship among both blocks and cells is represented by a cloud labelled “Cell *i* connection”.

**Figure 4:** Class relationship among datasets. Each dataset is represented by a rectangle labelled by the dataset name. In each rectangle, a class is highlighted by a silhouette labelled by the class name and numbers of its training and testing images. The classes of images containing similar-shaped objects are enclosed by polygons of different line colours, e.g., both the class vehicle in ENA24 and the class truck in CIFAR-10 contain images of various trucks, and thus, the two classes are enclosed in one polygon of brown lines.

**Figure 5:** A shallow regression tree. A regression tree is a stack of binary trees which conduct condition evaluations at nodes. A leaf node corresponds to a possible prediction yielded by the regression tree. A leaf node can be reached by walking along a path from the root to the leaf, and the “walk” means the input satisfies all conditions of nodes along the path. In this figure, different kinds of nodes are represented by rectangles painted by different colours, e.g., nodes involving $\dot{B}$ and $\ddot{B}$ are, respectively, denoted by red and blue rectangles, and the leaf nodes are represented by green nodes. The path between two nodes is denoted by arrows labelled “True” or “False”.

**Figure 6:** A deep regression tree. The meaning of graphical elements in this figure is the same as in Figure 5.

**Figure 7:** The normal cell found by NASRT. This figure is a concrete version of Figure 3, and hence, only the differences are described here. The output of a cell is indicated by an arrow with a dashed line whose colour is the same as the cell rectangle. Both operation outputs and block outputs are represented by arrows with solid black lines. Blocks are denoted by rectangles with dashed lines.

**Figure 8:** Examples of misclassified images from ENA24. This figure illustrates four misclassified image samples together with corresponding prediction results. The results associated with each image sample illustrate five top predictions yielded by NASRT, and both the predicted species names and the corresponding probabilities are represented by texts under the image sample. The probabilities are visualized by bars of different colours for visual discrimination. The ground-truth species are highlighted by green texts, and the erroneously predicted species are indicated by red texts. The animals of the ground-truth species in sample images are enclosed by red lines for enhancing the visibility of animals.

**Figure 9:** Misclassified northern raccoon images. The meaning of graphical elements in this figure is the same as in Figure 8.

**Figure 10:** Misclassified grey fox images. The meaning of graphical elements in this figure is the same as in Figure 8.

**Figure 11:** Misclassified bobcat images. The meaning of graphical elements in this figure is the same as in Figure 8.

**Figure 12:** Misclassified cottontail images. The meaning of graphical elements in this figure is the same as in Figure 8.

**Figure 13:** Examples of misclassified images from MCTI. The meaning of graphical elements in this figure is the same as inFigure 8.

**Figure 14:** Misclassified ocelot images. The meaning of graphical elements in this figure is the same as in Figure 8.

**Figure 15:** Misclassified red brocket deer images. The meaning of graphical elements in this figure is the same as in Figure 8.

**Figure 16:** Misclassified red fox images. The meaning of graphical elements in this figure is the same as in Figure 8.

**Figure 17:** Jetson X2. This figure illustrates an edge device named Jetson X2 in its working state.

**Table 1:** Search comparison.

Method	Para. (M)^†^	Test (sec.)^†^	GPU (MB)^†^	Time (GPU days)

NASRT (ours)	2.49	0.17	10.42	**0.27 ** ^†^
Resnet-18 [46]	11.19	**0.01**	44.81	Manual
DenseNet [47]	6.98	0.08	28.35	Manual
MobileNet-v2 [48]	**2.25**	0.05	**9.23**	Manual
PDARTS [24]	3.44	0.25	14.50	0.81^†^
SGAS [44]	4.42	0.27	18.54	0.97^†^
SETN [26]	4.63	0.27	19.31	1.08^†^
PNASNet [24]	4.28	0.17	17.53	225.00^‡^
MnasNet [45]	3.13	0.03	12.75	480.00^‡^
NASNet-A [22]	3.25	0.25	13.79	1800.00^‡^

^†^Obtained through our software or hardware or both; ^‡^cited from works of literature.

**Table 2:** Accuracy comparison based on ENA24.

Class	NASRT (ours)	Resnet-18 [46]	DenseNet [47]	MobileNet-v2 [48]	SGAS [44]	SETN [26]	PDARTS [24]
American black bear	96.93	**98.16**	95.09	95.71	93.87	96.32	96.32
American crow	98.06	**99.35**	**99.35**	92.90	98.71	96.77	**99.35**
Bird	**100.00**	**100.00**	**100.00**	97.14	**100.00**	91.43	**100.00**
Bobcat	**95.16**	**95.16**	93.55	**95.16**	90.32	80.65	93.55
Chicken	98.02	97.03	**99.01**	95.05	97.03	94.06	98.02
Coyote	96.61	**98.31**	**98.31**	96.61	**98.31**	**98.31**	96.61
Dog	96.83	**98.41**	97.62	96.83	96.03	97.62	96.83
Domestic cat	**96.55**	91.95	91.95	86.21	91.95	93.10	93.10
Eastern chipmunk	**100.00**	**100.00**	**100.00**	**100.00**	**100.00**	**100.00**	**100.00**
Eastern cottontail	95.24	92.06	**98.41**	87.30	92.06	87.30	90.48
Eastern fox squirrel	**96.72**	**96.72**	**96.72**	**96.72**	95.08	**96.72**	**96.72**
Eastern gray squirrel	96.43	**98.21**	96.43	96.43	96.43	94.64	**98.21**
Gray fox	94.67	96.00	**98.67**	90.67	92.00	88.00	89.33
Northern raccoon	94.12	94.12	**96.08**	88.24	94.12	92.16	92.16
Red fox	**97.26**	**97.26**	94.52	**97.26**	95.89	90.41	94.52
Striped skunk	**98.18**	96.36	**98.18**	92.73	92.73	96.36	92.73
Vehicle	**100.00**	**100.00**	**100.00**	**100.00**	**100.00**	95.45	95.45
Virginia opossum	98.48	99.24	**100.00**	98.48	**100.00**	99.24	99.24
White-tailed deer	98.36	98.36	**100.00**	96.72	96.72	95.08	96.72
Wild turkey	**100.00**	98.15	96.30	94.44	92.59	96.30	98.15
Woodchuck	**97.30**	**97.30**	**97.30**	**97.30**	94.59	**97.30**	**97.30**
Average	97.38	97.25	**97.50**	94.85	95.64	94.15	95.94

**Table 3:** Accuracy comparison based on MCTI.

Class	NASRT (ours)	Resnet-18 [46]	DenseNet [47]	MobileNet-v2 [48]	SGAS [44]	SETN [26]	PDARTS [24]

Agouti	**97.60**	95.21	96.41	95.81	96.41	89.82	92.81
Bird	98.61	97.92	97.92	99.31	**100.00**	98.61	**100.00**
Coiban agouti	**100.00**	**100.00**	**100.00**	**100.00**	99.61	98.06	**100.00**
Collared peccary	98.25	96.49	94.15	92.98	97.66	92.40	**98.83**
Opossum	**98.15**	94.44	96.91	96.30	**98.15**	93.21	97.53
European hare	97.48	89.92	96.64	96.64	96.64	**99.16**	94.96
Great tinamou	**99.56**	99.11	98.22	**99.56**	**99.56**	93.33	97.78
Mouflon	**99.77**	99.30	99.30	99.07	99.30	97.91	98.84
Ocelot	**89.47**	82.11	85.26	75.79	82.11	68.42	74.74
Paca	**100.00**	92.09	96.74	95.35	95.81	90.70	96.28
Red brocket deer	**96.59**	93.75	96.02	93.18	91.48	93.18	92.61
Red deer	**100.00**	**100.00**	99.80	**100.00**	**100.00**	99.61	**100.00**
Red fox	**95.60**	93.41	92.31	91.21	93.41	79.12	93.41
Red squirrel	**97.35**	93.81	94.69	93.81	94.69	88.50	87.61
Roe deer	**98.72**	98.29	98.29	98.29	98.29	96.58	98.29
Spiny rat	99.24	**100.00**	96.21	91.67	97.73	84.85	97.73
White-nosed coati	**99.57**	99.15	98.72	97.02	97.87	95.32	97.45
White-tailed deer	**99.75**	98.99	97.98	98.24	99.50	95.97	**99.75**
Wild boar	**99.71**	98.82	99.41	**99.71**	99.41	99.41	**99.71**
Wood mouse	**100.00**	**100.00**	**100.00**	**100.00**	**100.00**	**100.00**	**100.00**
Average	**98.27**	96.14	96.75	95.70	96.88	92.71	95.92

**Table 4:** Accuracies from Jetson X2.

ENA24 class	NASRT	MCTI class	NASRT

Black bear^†^	98.77	Agouti	95.21
Crow^†^	97.42	Bird	97.22
Bird	100.00	Coiban agouti	100.00
Bobcat	91.94	Collared peccary	99.42
Chicken	99.01	Opossum	98.15
Coyote	98.31	European hare	100.00
Dog	97.62	Great tinamou	98.67
Domestic cat	91.95	Mouflon	99.07
Chipmunk^‡^	100.00	Ocelot	78.95
Cottontail^‡^	92.06	Paca	99.53
Fox squirrel^‡^	96.72	Red brocket deer	94.89
Gray squirrel^‡^	98.21	Red deer	100.00
Gray fox	93.33	Red fox	93.41
Northern raccoon	94.12	Red squirrel	93.81
Red fox	95.89	Roe deer	99.15
Striped skunk	100.00	Spiny rat	96.21
Vehicle	100.00	White-nosed coati	99.57
Virginia opossum	100.00	White-tailed deer	99.24
White-tailed deer	93.44	Wild boar	99.41
Wild turkey	100.00	Wood mouse	100.00
Woodchuck	97.30	Average	98.23
Average	97.03		

^†^American species; ^‡^Eastern species.

## Data Availability

The codes used to support the findings of this study are available from corresponding authors upon request. Dataset ENA24 can be retrieved from https://lila.science/datasets/ena24detection. Dataset MCTI can be retrieved from https://lila.science/datasets/missouricameratraps.

## Supplementary Materials

Supplementary Materials A brief introduction of XGBoost and the detailed description of XGBoost hyperparameters can be found in Supplementary Materials.
